RETRACTED

# High dose of nimustine as an add-on treatment for small cell lung cancer with intracranial metastasis: A case report and literature review

**DOI:** 10.1097/MD.0000000000008218

**Published:** 2017-10-13

**Authors:** Wei Luo, Ya-lun Li, Ya Juan Chen, Qing Xiang, Hong Chen

**Affiliations:** a Department of Respiratory Medicine, The People's Hospital of Leshan, Leshan; b Department of Respiratory and Critical Care Medicine, West China Hospital, Sichuan University, Chengdu, Sichuan; c The First Affiliated Hospital of Chongqing Medical University, Chongqing, P.R. China.

**Keywords:** high dose, intracranial metastases, lung cancer, nimustine

## Abstract

**Rationale:**

Small cell lung cancer (SCLC) characterized by high degree of malignancy and rapid tumor progression. Intracranial metastases often appear at the time of the initial diagnosis or treatment. Besides of radiotherapy, chemotherapy is supposed to have limited effect.

**Patient concerns:**

A 66-year-old male had blurred vision and unsteady step with moderate headache, nausea, vomit.

**Diagnoses:**

The patient was diagnosed with SCLC with intracranial metastases.

**Interventions:**

High dose of nimustine (ACNU) (300 mg/m^2^) add to the regimen containing carboplatin and irinotecan.

**Outcomes:**

Although the patient suffered severe myelosuppression, the intracranial lesion almost disappeared and maintained half a year.

**Lessons:**

ACNU at a dose of 200 mg/m^2^ might be tolerable in combination with other chemotherapeutic drugs for the treatment of SCLC with intracranial metastases besides radiotherapy.

## 1 Introduction

Small cell lung cancer (SCLC) is the common type of lung cancer, which currently accounts for 13.6% of all lung cancers.^[1]^ In particular, it has been reported that 10% of patients with SCLC were found to have central nervous system (CNS) metastases at initial diagnosis, whereas 20% during therapy and 50% at autopsy.^[2,3]^ These metastases frequently impair the patient's activities of daily life and the median survival time is approximately 3.0 to 4.5 months.^[4]^ Whole-brain irradiation and corticosteroid therapy has been the standard treatment for SCLC patients with CNS metastases. Referring to chemotherapy, it was believed that water-soluble chemotherapeutic agents would be ineffective against brain tumors because inadequate doses of those agents are excluded by the barrier. Nimustine (ACNU) with the trait of **l**ipid-soluble at normal physiological pH levels has long been used in the treatment of malignant CNS lesions. Here we present a SCLC patient with brain metastases chose high dose of ACNU to treat the brain metastases.

## 2 Case report

The patient is a 66-year-old male pathologically diagnosed with SCLC in left lung 8 months ago. Systemic screening has been done and the clinical stage was determined to be limited disease, T_2_N_2_M0 (IIIA).^[5]^ The patient received standard chemotherapy with cisplatin and etoposide and refused to do prophylactic cranial irradiation. After 4 cycles of cisplatin and etoposide chemotherapy, the disease was evaluated as stable stage. However, before the fifth chemotherapy the patient had blurred vision and unsteady step with moderate headache, nausea, and vomiting. Brain MRI showed that brain metastases had emerged (Fig. 1); therefore, the disease was evaluated as progressive disease and extended disease. The patient stubbornly refused the whole-brain radiotherapy and chose high-dose ACNU chemotherapy as adding therapy. After he signed the consent form, ACNU was administered intravenously once daily (60 mg/m^2^/day) for consecutive 5 days adding to the regimen containing carboplatin and irinotecan. Three days after chemotherapy, this patient had suffered severe myelosuppression (agranulocytosis for 11 days, thrombocytopenia lasted for 12 months) (Figs. 2 and 3) and panniculitis. The bone marrow aspiration was applied twice and except the hemopoietic cell hypoplasia no metastasis was detected, whereas the platelet-associated antibody was negative. The patient was hospitalized in private rooms with ultraviolet air disinfection 3 times a day and received intravenous antibiotics including meropenem, vancomycin, and voriconazole. The granulocyte colony-stimulating factor and thromboietin were persistently applied for a period of time, whereas transfusion of plasma and platelet were administered when necessary. After taking these treatments, the patient gradually recovered. Two months later, the patient had taken the brain MRI and chest CT again. To our surprise, the encephalic lesion nearly disappeared whereas the lung lesion still stayed stable (Fig. 4). Seven months later the brain lesion recurred (Fig. 5) but it was smaller than the primary lesion and the patient received cranial irradiation. Now this patient survived nearly 2 years since being diagnosed without any obvious symptom except stubborn thrombocytopenia. The patient did not receive chemotherapy any more except best supportive care.

RETRACTED

**Figure 1:** The brain lesion before ACNU chemotherapy (red arrow).

**Figure 2:** The tendency of platelet 12 mo after the ACNU chemotherapy.

**Figure 3:** The tendency of white blood cell 12 mo after the ACNU chemotherapy.

**Figure 4:** The brain lesion almost disappeared 2 mo after the ACNU chemotherapy (red arrow).

**Figure 5:** The brain lesion recurred 7 mo later after the ACNU chemotherapy (red arrow).

## 3 Discussion

Usually the dose of ACNU administrated was <60 mg/m^2^/per cycle (1 day or consecutive days), or 2 to 3 mg/kg/per cycle. According to the literature review conducted in PubMed and Web of Science, we define high dose of ACNU as >200 mg/m^2^/per cycle, whereas the range varied from 200 to 1100 mg/m^2^/per cycle (Table 1). High dose of ACNU could be applied in acute lymphoblastic leukemia/acute myeloblastic leukemia (ALL/AML) for the purpose of destroying human immune system before bone marrow transplantation (BMT), glioblastoma, and malignant astrocytoma, however no such dose has been reported in SCLC with intracranial metastases. Izaki et al retrospectively evaluated early and long-term complications of an intensified ACNU or melphalan in 52 children with acute leukemia or non-Hodgkin lymphoma. ACNU was administrated at 200 mg/m^2^/d in consecutive 2 days followed by BMT. The author found both regimens were tolerable, whereas the ACNU-group had the high incidence of pulmonary complications.^[6]^ Wang et al compared ACNU-based to temozolomide-based chemotherapy in glioblastoma patients. The dose of ACNU was 90 mg/m^2^/per day in consecutive 3 days and both groups showed greater tolerability.^[7]^ The maximum dose of ACNU was 1100 mg/m^2^ reported by Nakagawa H, but the patient died soon.^[8]^ The middle dose 600,800 mg/m^2^ was also reported, but one died of intratumorous bleeding and the other of pulmonary fibrosis.^[9]^ Referring to the side effect of high-dose ACNU, hematological toxicity, neurotoxicity, and pulmonary complication are the major problems in the short and long term.^[7]^ In our case, we believe ACNU plays a major role in cranial lesion disappearing for 2 reasons. First, the cranial metastasis appeared after receiving 4 cycles of first-line chemotherapy and disappeared after the fifth chemotherapy containing ACNU. Second, in the fifth therapy regimen only ACNU has definite effect on cranial lesion for its special soluble trait. To determine whether ACNU is suitable for NSCLC with cranial metastasis, we need more researches. Besides using for intracranial malignant lesions, Isobe et al also reported that although grade 4 thrombocytopenia was observed in 13% of patients, applying relative high dose of ACNU in a short period, 238 mg/m^2^ in 39.7 days, provided a practical and well-tolerated regimen that was active for irinotecan-refractory SCLC.^[10]^ As a conditioning regimen without BMT support, ACNU at a dose of 200 to 400 mg/m^2^ has been reported to be tolerable in combination with other chemotherapeutic drugs.^[6]^ The total dose of ACNU applied in this patient was 300 mg/m^2^, so we recommend <200 mg/m^2^ might be a safe dose to avoid severe myelosuppression. To sum up, for SCLC with intracranial metastases, no more than 200 mg/m^2^ of ACNU as an add-on treatment to standard chemotherapy might be a safe and effective choice besides radiotherapy.

RETRACTED

**Table 1:** Studies using high dose of ACNU.
